# Effect of Algoplaque Hydrocolloid Dressing Combined with Nanosilver Antibacterial Gel under Predictive Nursing in the Treatment of Medical Device-Related Pressure Injury

**DOI:** 10.1155/2022/9756602

**Published:** 2022-07-11

**Authors:** Chunxiu Li, Hongmei Chen, Guanghui You

**Affiliations:** ^1^Department of Neurosurgery, Chongqing Qijiang District People's Hospital, Chongqing 401420, China; ^2^Department of Endocrinology, Chongqing Qijiang District People's Hospital, Chongqing 401420, China; ^3^Department of Gastroenterology, Chongqing Qijiang District People's Hospital, Chongqing 401420, China

## Abstract

It was aimed at the clinical value of predictive nursing and Algoplaque hydrocolloid dressing (AHD) combined with nanosilver antibacterial gel in treating medical device-related pressure injury (MDRPI). 100 patients, who underwent surgery in Chongqing Qijiang District People's Hospital from February 2019 to February 2020, were selected as the research objects and were randomly divided into the experimental group (50 cases) and the control group (50 cases). For the characterization test, a nanosilver antibacterial gel was created first. Patients in both groups received predictive nursing, but those in the experimental group received AHD and nanosilver antibacterial gel, and those in the control group received gauzes. MDRPI incidence, pressed skin injury severity, comfort level, clothing changes, nursing satisfaction, and other factors were all compared. The particle size of the nanosilver gel was 45-85 nm, with a relatively homogeneous distribution with the medium size, according to the findings. The incidence of MDRPI in the experimental group was lower than that in the control group significantly (6% vs. 30%, *P* < 0.05). The degree of injury of pressured skin in the experimental group was milder than that in the control group (*P* < 0.05), the degree of comfort and nursing satisfaction was higher in the experimental group than in the control group (*P* < 0.05), and dressing change count was lower than that in the control group (*P* < 0.05). In the treatment of MDRPI, predictive nursing and AHD using nanosilver antibacterial gel showed high clinical application value.

## 1. Introduction

Various complex medical technologies emerge and are widely used in clinical practice as medical technology continues to develop and progress. Medical device-related pressure injury (MDRPI) occurs when modern medical equipment are employed in clinical settings [1, 2]. With the deepening researches, the relevant theories of MDRPI are accepted and recognized clinically. Clinical studies have shown that the appearance of skin injury caused by medical devices is generally the same as that of medical devices, and the most common injury sites include the head, face, neck, and limbs [3]. In recent years, most of the reports on MDRPI are reported in the intensive care unit (ICU), of which 1/3 of the skin injury is caused by medical devices. MDRPI often results in adverse complications such as infection, which influence the prognosis and postrecovery greatly [4–6]. At present, domestic researches mostly focus on MDRPI caused by a certain type and a certain factor, suggesting a lack of prospective and multicenter research [7].

Predictive nursing is guided by holistic nursing, with prevention first and then treatment. In its clinical application, it has shown significant curative effect in preventing and controlling complications [8, 9]. Some scholars have applied the predictive nursing to cardiopulmonary bypass surgery, which turns passive work into active work, shortening the operation time and reducing the incidence of complications effectively [10]. In addition, predictive nursing is carried out for preventive care on the grounds of the patient's condition, so that human resources are optimally prepared before the condition changes, thus highly improving the quality of nursing [11]. All in all, predictive nursing is an effective way to promote the effectiveness, standardization, and refinement of nursing. It can not only greatly prevent nursing defects but also improve the preventability and controllability of nursing, having a high clinical application value [12].

Relevant clinical studies have shown that the incidence and severity of MDRPI in patients using Algoplaque hydrocolloid dressing (AHD) are significantly higher than those in control patients [13]. That may be because the AHD is a semipermeable hydrogel dressing that can adhere to the skin surface, absorb exudate 30 times of its own mass, and swell to form a mild and moist gel filling layer. As a result, the direct stimulation of moisture to the skin is decreased, and the stressed skin is protected. On the other hand, it can successfully increase blood circulation in the pressurized skin and relieve congestion in the patient's pressurized area. AHD has a certain thickness with a smooth and soft surface, which can effectively buffer the pressure and other damage to the skin, so as to prevent and reduce the pressure injury of the patient's skin [14]. In clinical treatment, the long-term use of medical devices will cause patients to experience adverse symptoms such as skin ulceration and itching. AHD can be gently and safely sticked on the skin, protecting the local skin and relieving the discomfort of the patient effectively [15]. With the advancement of science and the rapid development of nanotechnology over time, nanosilver has emerged and has shown more advantages apart from the effect of silver itself [16]. Nanosilver gel is a gel made of nanosilver, and it is mostly used in wounds. The unique physical features of gel will allow nanosilver to work continuously and efficiently limit bacterial growth and proliferation. It can also cause bacterial proteins to denaturize, which aids in sterilisation [17].

Under the predictive nursing, the effect of AHD combined with nanosilver antibacterial gel was discussed in the treatment of MDRPI. This work was aimed at laying a foundation for promoting the compliance of patients and improving the treatment outcomes.

The paper's organization paragraph is as follows: the materials and methods is presented in section 2.  Section 3 discusses the experiments and results.  Section 4 consists of the conclusion section of the proposed work. Finally, in Section 5, the research work is concluded.

## 2. Materials and Methods

### 2.1. Research Objects

The research subjects were 100 patients who underwent surgery at Chongqing Qijiang District People's Hospital between February 2019 and February 2020. There were 55 male patients and 45 female patients, with an average age of 42.3 ± 10.3 years old. The patients were randomly divided into the experimental group with 50 cases and the control group with 50 cases as well. Inclusion criteria were as follows. The age of patients should be ≥12 years old. There was no pressure ulcer or skin injury or scar tissue prior to surgery or the use of medical equipment. The surgery was the first surgery during hospitalization, and the estimated operation time was ≥2 hours. The criteria for exclusion are stated below. During the procedure, the patients were given either local infiltration an aesthetic or nerve block anesthesia. The patients had severe skin disorders or conditions that interfered with skin observation. If the surgery was an emergency surgery, the patient was also excluded. All the patients signed informed consents, and all studies here conformed to the medical ethics.

### 2.2. Preparation Method of Nanosilver Mixture Solution

400 mg of silver nitrate was added to 1 L of distilled water or ultrapure water, and the mixture was stirred well. Under magnetic stirring (1600 r/min), 300 m of povidone K-30 or 300 mg of poloxamer 407 was added. After stirring evenly, 300 mg of trisodium citrate was also added. Then, the ultraviolet lamp was turned on. With the reaction under the irradiation of the ultraviolet lamp and magnetic stirring for 4-5 hours, the nanosilver mixture could be obtained. The obtained liquid was centrifuged, and then, the supernatant was discarded. The remains were diluted with distilled water or ultrapure water and then were centrifuged again, and these steps were repeated twice. Finally, the nanosilver precipitate obtained after centrifugation was dried, and an appropriate amount of nanosilver solution was weighed to prepare a 240 *μ*g/mL nanosilver stock solution.

Characterization test of the nanosilver solution was performed. In the scanning electron microscope (SEM) experiment, 1-2 drops of sample solution were added dropwise to a clean glass slide and dried in a constant temperature oven at 50°C, and then, the surface was gold-plated. The microstructure of the nanosilver solution was observed on an ultra-high-resolution field emission SEM. The main parameters selected were 10 KV high pressure, high vacuum mode, and secondary electron mode. In X-ray powder diffraction experiment, the nanosilver powder obtained by drying was used, the scanning angle was 10°-90°, and the Cu target was taken as the X-ray generating device.

### 2.3. Preparation of Nanosilver Antibacterial Gel

15 mL of distilled water was added into a 50 mL beaker and 200 *μ*L of glacial acetic acid, and then, 2,000 *μ*L of the prepared nanosilver solution was added to the distilled water in turn. 600 *μ*L of glycerol was also added and stirred until it was completely dissolved. After that, 0.42 g of chitosan was added, stirred evenly, and left overnight. The mixture was fully swelled, and the air bubbles were removed. Finally, 2 mL of sodium bicarbonate solution with a concentration of 1 mol/L was added dropwise into the beaker. Distilled water was added dropwise after stirring evenly to prepare a 20 mL of sol system, which was allowed to stand for a few days to form a gel.

Characterization of the nanosilver gel was also performed. An appropriate amount of the prepared chitosan wet gel was put into a desiccator for drying at room temperature. When the weight of the gel no longer changed, a small amount of dry gel sample was taken out and pulled apart; then, the surface was gold-plated. The microstructure of the gel section was observed on the ultra-high-resolution field emission SEM. The selected parameters included the high pressure of 10 KV, high vacuum mode, and secondary electron mode, and the magnification was 5000 times.

### 2.4. Nursing Methods

Patients in both groups were treated with the predictive nursing, as the specific methods were described as follows.

To begin, the patients are seen and assessed before to surgery. The circulating or scrub nurse did a preoperative visit and assessment the day before the surgery after receiving news of the surgery. The medical records of the patient, as well as numerous examination indicators, were thoroughly checked, and anomalous indicators were noted. The nurse learned about the patient's medical history, described the intraoperative precautions, and assessed the patient's skin condition. Second, there are critical point shifts. The circulating or scrub nurse fed the collected abnormal conditions back to the on-duty nurses timely, and the key points could be highlighted at the morning shift. Thus, the medical staff would pay more attention to the abnormal conditions. Third is the reevaluation on the day of the surgery. On the day of the surgery, reevaluation was carried out according to the results of the skin evaluation of the preoperative visit, especially the abnormal parts needed to be paid more attention. Fourthly, the operation time was estimated according to the anesthesia method, surgical position, surgical method, and intraoperative external force. Then, a comprehensive evaluation was made, and corresponding surgical measures were taken. Fifthly, the corresponding nurse mode should be adopted depending on the patient's own diseases. For example, the blood circulation of the peripheral end of the foot of the diabetic patient was not good. It is also important to keep the foot warm while doing postural nursing. Sixth, to avoid alterations in the microenvironment around the skin, the surrounding skin was kept clean and dry. Seventhly, the use of medical devices should be reduced, and the prevention should be strengthened during surgery. With the surgical plan for the patient, the number of medical equipment used should be reduced as much as possible without affecting the curative effect. Eighthly, the key observations were implemented on key parts. Before the surgery, the skin of the pressured area was checked again, especially the skin pressured by the medical devices. The parts with higher risk were marked and focused on with close observation intraoperatively. Ninthly, awareness of prevention should be raised and continuing education should be strengthened.

Apart from the above-mentioned nursing measures, the patients in the experimental group used AHD and nanosilver gel to protect the key parts, especially the areas would be pressured by medical devices. The medical equipment could then be worn after that. Gauze was used to cover the important sections for protection in the control group.

### 2.5. Observation Indicators

The incidence of MDRPI, the degree of injury to the pressured area, comfort level, nursing satisfaction, and more indicators were statistically analyzed between the two groups. The specific evaluation criteria for the degree of injury and comfort level are shown in Tables 1 and 2, respectively.

### 2.6. Statistical Analysis

All data analyses were completed by SPSS19.0 software. The measurement data were expressed as mean ± standard deviation, and the test method was the independent sample *t* test. The enumeration data were expressed as frequencies, and the comparison between groups was done by chi-square test. *P* < 0.05 meant the difference was statistically significant.

## 3. Results

### 3.1. General Information of Patients

The general data of patients in the two groups are shown in Table 3. The experimental group included 26 male cases and 24 female cases, having an average age of 33 ± 11.3 years old. In the control group, there were 31 male patients and 19 female patients, and the average age of the patients was 36 ± 9.96 years old. No significant difference was discovered in the general data such as gender, age, department, and surgical position between the two groups, which showed the comparability.

### 3.2. Comparison of the Incidence of MDRPI between the Two Groups

The incidence of MDRPI was compared between the two groups, and the comparison results are shown in Figure 1. There were 3 patients with MDRPI in the experimental group (6%) and 47 patients without MDRPI (94%). MDRPI was found in 15 cases (30%) in the control group, but MDRPI was not found in the remaining 35 cases (70%). The differences between groups were of statistical significance (*P* < 0.05).

### 3.3. Comparison of the Degree of Skin Injury in the Two Groups

The comparison results of the degree of skin injury in the two groups of patients are shown in Figure 2. 1 (2%), 1 (2%), and 1 (2%) patient got mild, moderate, and severe skin injury, respectively, in the experimental group. In the control group, there were 4 (8%), 8 (16%), and 3 (6%) patients had mild, moderate, and severe skin injury, respectively. The differences between the groups were deemed statistically significant by the researchers (*P* <0.05).

### 3.4. Comparison of Comfort Level and Dressing Changes between the Two Groups

The comfort level and dressing changes of patients were compared between two groups, as shown in Figure 3. In the experimental group, the number of patients whose comfort levels were comfortable, less comfortable, general, and uncomfortable was 45 (90%), 2 (4%), 2 (4%), and 1 (2%), respectively. The number of patients in the control group whose comfort level was comfortable, less comfortable, average, and uncomfortable was counted to be 12 (24%), 15 (30%), 15 (30%), and 8 (16%), respectively. The differences between groups were also statistically significant (*P* < 0.05). The number of dressing changes in the experimental group was 0.5 ± 0.08 times, and that in the control group was 4.4 ± 0.22 times, showing a statistically significant difference as *P* < 0.05.

### 3.5. Comparison of Nursing Satisfaction of Patients in the Two Groups

The comparison of nursing satisfaction between the two groups is shown in Figure 4. It was found that, in the experimental group, the number of patients whose nursing satisfaction was satisfied, less satisfied, and unsatisfied was counted as 36, 12, and 2, respectively. The total satisfied rate for nursing was 72% in the experimental group. There were 11 satisfied patients, 15 less satisfied patients, and 24 unsatisfied patients in the control group, and the total satisfied rate was 22%. With the comparison between two groups, the nursing satisfaction of the experimental group was higher than that of the control group significantly (*P* < 0.05).

### 3.6. SEM Results of Nanosilver Antibacterial Gel

The SEM results of nanosilver are shown in Figure 5. The particle size of the nanosilver antibacterial gel prepared in this research was 45-85 nm, and the particle size was medium and distributed uniformly. It not only avoided the reduction of antibacterial activity due to excessive particle size but also avoided increased cytotoxicity for the too small particle size. Besides, it could also be observed that the nanosilver particles were wrapped by polymer materials.

## 4. Discussion

Clinical studies have indicated that MDRPI can be induced by a range of factors, including the material qualities of the device, difficulty helping or immobilising the patient's body, or persistent pressure release in the same location [18]. Patients' comfort levels will be substantially impacted with the onset of MDRPI, leading in decreased compliance and, as a result, treatment. If no appropriate therapy is given after the emergence of MDRPI, it can lead to infection and inflammation, which can have a negative impact on the disease's prognosis and treatment. Clinical research data suggest that MDRPI accounts for 34.5% of all pressure injuries, so its incidence is quite high [19]. If effective preventive intervention measures can be taken, it is of great significance to improve the curative effect, reduce the pain, and improve the compliance of patients.

The predictive nursing is also called advanced nursing, which refers to the nursing staff analyze and predict the specific situation of the patient as well as possible nursing problems before and during the nursing process, utilizing nursing knowledge. Thereby, the nursing focuses can be determined, and the preventive measures can be taken in advance to minimize the pain and accidents of patients. It is a nursing method change from passive to active [20–22]. Compared with traditional nursing methods, predictive nursing is more systematic, comprehensive, and individualized and has more advantages [23]. Some scholars have applied predictive nursing to the transfer nursing of emergency patients and patients with severe traumatic brain injury, which has greatly shortened the transfer time, reduced the incidence of transfer accidents, and improved nursing safety [24].

One of the most widely utilized clinical approaches for treating and preventing pressure injuries is AHD. Traditionally, materials such as gauze were used to treat antipressure skin injuries [25]. Gauze has been shown in clinical investigations to have flaws like hygroscopicity, poor air permeability, and easy displacement, all of which contribute to a poor fit between the skin and the medical device. The local skin is prone to fibrous impressions and even problems such as flush and erosion with long-term gauze use. In addition, due to the hygroscopicity of gauze, it increases the irritation of the patient's skin for moisture, so that it is often necessary to replace the gauze every 1-2 days. The workload of the nursing staff is increased, but also, damage would be caused to the skin by pulling the gauze repeatedly [26]. In comparison, the AHD can be safely attached to the skin, and it has good self-adhesiveness. It can protect the skin and absorb exudates effectively; meanwhile, its softness, a certain thickness, and other advantages can make it reduce and relieve pressure effectively [27]. Nanosilver gel is a kind of skin gel commonly used in clinical practice. Compared with other external drugs, nanosilver gel can reduce exudation obviously, improve wound healing rate, and shorten wound healing time. Thereby, the formation of scars is also reduced, improving the quality of healing [28, 29]. Some scholars have used nanosilver antibacterial gel combined with AHD in the treatment of unstageable pressure ulcers, and a higher cured rate was achieved than using AHD alone [30]. In general, nanosilver antibacterial gel has a high clinical application value in the treatment of skin wounds.

In this research, 100 patients were chosen as the research objects, as they were subjected to surgery in Chongqing Qijiang District People's Hospital from February 2019 to February 2020. All these patients were cared for with the predictive nursing after surgery. Nanosilver antibacterial gel was also prepared independently and was characterized by SEM. During the nursing procedure, the experimental group's patients were treated with AHD mixed with nanosilver antibacterial gel as pressed skin dressings, whereas the control group's patients were treated with gauzes. Afterwards, the incidence of MDRPI, the degree of skin injury, comfort level, nursing satisfaction, and more indicators were compared between the two groups. It was proved from the results that the nanosilver antibacterial gel prepared had uniform and moderate particle size with good quality. The incidence of MDRPI in the experimental group was remarkably lower, the degree of skin injury was slighter, and the comfort level and nursing satisfaction were higher significantly.

## 5. Conclusion

The nursing impact of nanosilver antibacterial gel mixed with AHD on pressed skin in the predictive nursing mode was investigated in this study. All the incidence of MDRPI, the degree of injury, comfort level, and nursing satisfaction were improved notably. MDRPI incidence, pressed skin injury severity, comfort level, clothing changes, nursing satisfaction, and other factors were all compared. The nanosilver antibacterial gel created had a homogeneous particle size, moderate particle size, and good quality, according to the findings. It was suggested that the combination of predictive nursing, AHD, and nanosilver antibacterial gel had a high clinical application value in the treatment of MDRPI.

## Figures and Tables

**Figure 1:** Comparison of the incidence of MDRPI between the two groups. Note: ^∗^*P* < 0.05 was obtained compared with the data of the control group.

**Figure 2:** Comparison of the degree of skin injury in patients in the two groups. Note: ^∗^*P* < 0.05, compared with those of the control group.

**Figure 3:** The comfort level and number of dressing changes of patients in the two groups. Note: ^∗^*P* < 0.05, which were compared with those in the control group.

**Figure 4:** Comparison of nursing satisfaction of patients between two groups. Note: ^∗^*P* < 0.05 compared with those of the control group.

**Figure 5:** SEM results of nanosilver antibacterial gel.

**Table 1:** Evaluation criteria for the degree of injury in the pressured area.

Degree of injury	Symptom description
Mild	The skin of the pressure area was sore, slightly painful, and without induration; the symptoms were relieved after the pressure was relieved.
Moderate	Redness, swelling, and induration occurred in the skin at the pressured area, with obvious pain after touching and no relief after the pressure was relieved.
Severe	Skin damage and ulceration appeared in the area of pressure.

**Table 2:** Evaluation criteria for comfort level of patients.

Comfort levels	Symptom description
Comfortable	No discomfort in the pressured area
Less comfortable	Slight discomfort in the pressured area
General	Pain after pressure
Uncomfortable	Severe pressured pain

**Table 3:** General data of patients in the two groups.

Items	Experimental group (50 cases)	Control group (50 cases)	*P*
Gender			
Male	26	31	0.51
Female	24	19	0.48
Age			
Departments	33 ± 11.3	36 ± 9.96	1.10
Otorhinolaryngology	05	06	1.20
Thoracic surgery	07	09	1.11
Neurosurgery	11	08	0.88
Obstetrics	04	06	0.93
Orthopedics	23	21	0.64
Injury areas			
Face	08	11	1.13
Nose	09	10	1.06
Ears	12	11	1.33
Chests	16	14	0.97
Upper arms	03	04	0.68
Knees	02	01	0.72
Surgical positions			
Supine position	19	17	0.81
Prone position	17	18	0.92
Lateral position	14	15	0.77
Anesthesia			
General anesthesia	26	30	0.55
Intraspinal anesthesia	24	20	0.63

## Data Availability

All data, models, and code generated or used during the study appear in the submitted article.
